# The Mental Health and Grade Point Average among College Students from Lower Socioeconomic Status Based on Healthcare Data Analysis

**DOI:** 10.1155/2021/2378202

**Published:** 2021-11-30

**Authors:** Xue Dong, Kaige Yang, Ruxin Zhang, Yuecheng Lv

**Affiliations:** ^1^Mental Health and Counseling Center, Student Affairs, Shaanxi University of Science & Technology, Xi'an, Shaanxi, China; ^2^College of Education, Shaanxi University of Science & Technology, Xi'an, Shaanxi, China; ^3^Department of Economics and Management, Xi'an University of Technology, Xi'an, Shaanxi, China; ^4^School of Materials Science & Engineering, Shaanxi University of Science & Technology, Xi'an, Shaanxi, China

## Abstract

This study evaluated the mediating role of social support in the relationships between mental health and academic achievement and used a sample of 640 college students from lower socioeconomic status (LSES) compared to 501 from higher socioeconomic status (HSES) in China. Self-report measures of depression, anxiety, Internet addiction, self-esteem, perceived social support, and grade point average (GPA) were measured online. Group differences were examined with Chi-square analyses. *Results*. (1) There were significant differences in mental health, academic achievement, and social support between LSES and HSES. (2) Anxiety, depression, and Internet addiction were significantly negatively correlated with academic achievement; self-esteem and social support were significantly positively correlated with academic achievement. (3) Social support has a mediating role between mental health and academic achievement. These results proved that it is necessary to pay more attention to their mental health and develop social support to improve their academic achievement for LSES students. Previous studies have paid little attention to the LSES students, but these students are more prone to psychological problems. Therefore, this study focuses on the LSES students.

## 1. Introduction

Academic achievement has always been an important aspect of life for college students. Grade point average (GPA) is one of the most frequently used measures in academic achievement research and is typically regarded as one of the most important indicators of a student's success at university, potentially influencing both financial aid in the short term and career prospects in the long term. An extensive literature showed that GPA was associated consistently with numerous psychological outcomes, such as depression, anxiety, psychological distress, self-esteem, and problem behaviors among adolescents [1–5]. For instance, depression and anxiety predict impairment of academic achievement among a sample of 5,689 college students [6]. However, these associations have not been examined among students with financial difficulties, a group that may be at elevated risk for mental health disorders.

A highly visible cultural variable that has tended to differentiate rich and poor is socioeconomic status (SES). The definition of SES incorporates parental income, parental education, and parental occupation as the three main indicators of SES [7]. SES is generally considered to be one of the most important factors affecting the development of young people in all aspects, generally higher social capital status often means life success. In recent years, the number of college students coming from LSES has been increasing year by year in China. According to the theory of the family investment model, families from HSES have a stronger ability to devote themselves to education, and their children tend to perform better in school [8]. Families from LSES are less likely to devote to education, and children are more likely to develop psychological and behavioral problems as teenagers, such as depression, anxiety, and Internet addiction [9]. The factors of economic hardship will affect students' mental health and further affect students' academic achievement [10]. Although prior research has focused on different socioeconomic groups, there are relatively little research studies on the relationship between mental health and academic achievement of students from LSES.

In addition, some researchers have found that social support can effectively predict college students' academic achievement. Social support is a kind of helping function provided by friends, family, and significant others, which can provide instrumental, informational, or emotional assistance. Perceived social support is closely related to various social functions and mental health, such as it predicts psychological adaptability, reduces suicide risk and loneliness, relieves depression, anxiety, and physical illness, and reduces the risk of academic failure and dropout [11]. Social support can predict academic achievement and is an important factor to promote academic achievement [12]. One path analysis suggests that self-esteem fully mediates the relationship between social support and academic achievement in a sample of 262 college students in China [13]. Less family support and more parental conflicts have the most significant impact on the lowest academic achievement of female college students [14]. College students with lower social support were more likely to experience depressive symptoms relative to students with higher social support [15]. Furthermore, social support may be an effective mediator between psychological quality and academic achievement, and the underlying mechanism still needs further study.

The study aims to examine the underlying mechanism among social support, mental health, and GPA among college students from LSES. Based on the previous literature, we hypothesized that (1) the mental health of students from LSES is negatively related to GPA, (2) social support has a positive effect on GPA, and (3) social support mediates the relationships between mental health and GPA (Figure 1).

## 2. Methods

### 2.1. Participants and Procedure

The cross-sectional study was conducted during May and June 2020 and 1156 participants were recruited from one college in China. The data of 1156 participants (628 or 55% males and 513 or 45% females) aged 15–28 (20.24 + 1.34, mean + SD) years were analyzed in the current study. Participants in the study were divided into LSES and HSES groups based on certain criteria. Participants 640 (56.1%) with LSES were identified by the Chinese government according to the standard of $390 income yearly, parents' education (mother and father's), and parents' occupations. Participants 501(43.9%) were the HSES group identified by the parents with college graduates and postgraduate degrees and with yearly incomes of $1500 or more. Informed consent was obtained from all subjects involved in the study. The research proposal was approved by the Ethical Committees of Shaanxi University of Science & Technology.

### 2.2. Measures

The survey assessed symptoms of four types of mental health-related disorders and problems: depression, anxiety, Internet addiction, and low self-esteem. We focused on these conditions because they are some of the most prevalent in college students. The overall past year incidence of anxiety was 26.60% and depressive emotions were detected in 21.16% of the college students in 2020 [16]. The pooled detection rate of Internet addiction was 11% among college students in China in 2018 [17]. LSES students showed high materialism tendencies to compensate for self-esteem in China [18].

#### 2.2.1. Internet Addiction Test (IAT)

IAT (1998) has 20 items rated on a six-point Likert scale, ranging from 0 (Not at all) to 5 (Always), to assess the impact of Internet use on daily lives. A higher score indicates a higher degree level of Internet addiction: 0–30 points are considered normal, 31–49 points are mild, 50–79 points are moderate, and 80–100 points are severe level of Internet dependence. A cut-off 50 or higher score is characterized as problematic Internet use and a score of 80 or higher as pathological use [19, 20]. Psychometric studies have indicated that high reliability, validity, and internal consistency [21].

#### 2.2.2. Beck Depression Inventory Second (BDI-II)

BDI-II consists of 21 items addressing symptoms of depression in the previous two weeks (e.g., hopelessness, irritability, guilt, fatigue, and weight loss) [22], each of which has four self-evaluative statements scored from 0 = minimal depression to 3 = severe depression. Depression classification criteria: 0–13 indicate no depression, 14–19 indicate mild depression, 20–28 indicate moderate depression, and 29–63 indicate severe depression. The higher the score, the higher the severity of depression. The BDI-II scale has been proven to have good internal reliability, consistency, and validity [23].

#### 2.2.3. State-Trait Anxiety Inventory (STAI)

STAI is a commonly used measure of trait and state anxiety. It has 20 items for assessing trait anxiety and 20 for state anxiety. State anxiety items include “I am tense; I am worried” and “I feel calm, I feel secure.” Trait anxiety items include “I worry too much over something that does not matter” and “I am content; I am a steady person.” All items are rated on a 4-point scale (e.g., from “Rarely” to “Almost Always”). Half of the items were reverse coded so that higher scores indicated greater anxiety. Items were summed to create a composite anxiety score with a possible range of 20–80 [24].

#### 2.2.4. Rosenberg Self-Esteem Scale (RSES)

RSES includes 10-items rated on a 4-point Likert scale (1 strongly disagree to 4 strongly agree) and was designed to measure an individual's self-esteem and self-acceptance. A sample item is “On the whole, I am satisfied with myself.” Higher scores represent higher self-esteem [25].

#### 2.2.5. Multidimensional Scale of Perceived Social Support (MSPSS)

MSPSS has 21 items with a 7 point response format (1 = very strongly disagree; 7 = strong and agree). It is comprised of three subscales, each addressing a different source of support: family support, friend support, and significant other support. MSPSS has good internal and test-retest reliability as well as moderate construct validity [26].

#### 2.2.6. Academic Achievement

Academic achievement was the main dependent variable in this study. Academic achievement was assessed through self-reported cumulative GPA ranging from 1.50 to 5.00 for the previous semester which was used as a continuous variable.

### 2.3. Statistical Analyses

In the current study, statistical analyses were performed using SPSS 19.0 and AMOS 21.0 software. To examine the difference in the association between the variables, participants were split into 2 groups according to LSES and HSES. Structural equation modeling (SEM) was then used to test the structural model and verify the relationship between variables. Bootstrap procedure was used to test the mediating effect of social support based on 5000 samples. The statistical significance was set at *p* < 0.05 (two-tailed).

## 3. Results

### 3.1. Comparing Clinical Variables between LSES and HSES

There are significant differences between the LSES group and the HSES group in state anxiety, trait anxiety, self-esteem, depression, and Internet addiction, significant other support, family support, friend support, and GPA (*p* < 0.05). Specifically, the LSES group score is higher than the HSES group in terms of state anxiety, trait anxiety, depression, and Internet addiction; HSES score is higher in self-esteem, significant other support, family support, friend support, and GPA than the LSES group (Table 1).

### 3.2. Pearson's Correlation Coefficients between Clinical Variables in Whole Samples

Pearson's correlation was used to present the descriptive and correlations among depression, state anxiety, trait anxiety, self-esteem, depression, Internet addiction, social support, and GPA. State anxiety (*r* = −0.619, *p* < 0.01), trait anxiety (*r* = −0.597, *p* < 0.01), depression (*r* = −0.570, *p* < 0.01), and Internet addiction (*r* = −0.413, *p* < 0.01) were significantly negatively related to GPA. Additionally, self-esteem (*r* = 0.466, *p* < 0.01), significant other support (*r* = 0.617, *p* < 0.01), family support (*r* = 0.609, *p* < 0.01), and friend support (*r* = 0.550, *p* < 0.01) were significantly positively correlated to GPA (Table 2). These relationships have offered the statistical foundation to examine our hypothesized mediation model.

### 3.3. Mediation Effect: Social Support as the Mediator

The hypothesized model showed good fit to the data. As shown in Figure 2, state anxiety (*β* = −0.238, *p* < 0.001), trait anxiety (*β* = −0.085, *p* < 0.05), depression (*β*=−0.085, *p* < 0.01), and Internet addiction (*β* = −0.099, *p* < 0.001) had a negative and significant effect on GPA. Significant other support (*β* = 0.153, *p* < 0.001), family support (*β* = 0.092, *p* < 0.01), friend support (*β* = 0.144, *p* < 0.001), and self-esteem (*β* = 0.083, *p* < 0.001) had a positive and significant effect on GPA.

Additionally, state anxiety (*β* = −0.213, *p* < 0.001), trait anxiety (*β* = −0.291, *p* < 0.001), depression (*β* = −0.107, *p* < 0.001), and Internet addiction (*β* = −0.141, *p* < 0.001) had a negative and significant effect on significant other support. Self-esteem (*β* = 0.085, *p* < 0.01) had a positive and significant effect on significant other support.

State anxiety (*β* = −0.179, *p* < 0.001), trait anxiety (*β* = −0.215, *p* < 0.001), depression (*β* = −0.262, *p* < 0.001), and Internet addiction (*β* = −0.081, *p* < 0.01) had a negative and significant effect on family support. Self-esteem (*β* = 0.083, *p* < 0.01) had a positive and significant effect on family support.

State anxiety (*β* = −0.115, *p* < 0.01), trait anxiety (*β* = −0.102, *p* < 0.05), depression (*β* = −0.280, *p* < 0.001), and Internet addiction (*β* = −0.064, *p* < 0.05) had a negative and significant effect on friend support. Self-esteem (*β* = 0.125, *p* < 0.01) had a positive and significant effect on friend support.

To test the mediating effect of social support, the Bootstrap method was used to test mediating effect. The 95% confidence interval of all mediation effects does not include 0 (*p* < 0.05), so all mediating effects were validated (Table 3).

## 4. Discussion

### 4.1. Mental Health of LSES College Students

The study showed that the scores of state anxiety, trait anxiety, depression, and Internet addiction were higher in the LSES group compared with the HSES group. While the scores of self-esteem in the LSES group were lower than the HSES group. Consistent with previous research, we confirmed that SES can significantly predict adolescents' mental and behavioral problems. For instance, LSES had a great impact on adolescents' mental health and behavioral development of adolescents among 1337 adolescents in 13 middle schools [27]. SES had a significant negative predictive effect on college students' social anxiety, confirming the influence of SES on mental health [28]. Compared with ordinary college students, there were more rates of depression symptoms among LSES college students [29], indicating that long-term LSES was the main factor for young people's mental health problems [30]. Particularly, external factors such as heavy economic pressure and living difficulties can cause psychological problems such as tension, anxiety, and low self-esteem for students with LSES, resulting in higher psychological pressure than other groups of students [31, 32]. The conclusions of the study put forward that the mental health of LSES students was worse than other groups, which requires special attention.

### 4.2. Relationship between Impacts of Mental Health on the Academic Achievement of LSES College Students

The results indicated that the GPA of the LSES group was lower than the HSES group. We found that state anxiety, trait anxiety, depression, and Internet addiction had a negative and significant impact on GPA, and self-esteem had a positive significant impact on GPA. The results were consistent with other studies that mental health had a significant predictive effect on academic achievement. Specifically, there was a significant correlation between high anxiety and low academic achievement among college students [33]. The negative impact of depression on the academic productivity of college students and most students with good family support perform better in academics than the ones with low-income family support [34]. Students with greater emotional distress also report worse academic achievement, the relationship of depression with self-reported GPA was mediated by the frequency of failed exams [35]. The results may be due to participants with severe depression who are more likely to fail the exam. Moreover, we observed Internet addiction was negatively correlated with academic achievement. Indulging on the Internet may lead to loneliness, depression, and other unhealthy psychological conditions; internet-addicted medical students scored significantly poorly in their exams, so it affects academic achievement [36].

Concerning the impact of the mental health of students with LSES on their academic achievement, previous research has also supported the conclusions of this study. The HSES students will devote more to learning; parents of the HSES can provide their children with better material conditions and choose superior educational resources to ensure their children's academic achievement [37]. HSES can significantly positively affect mathematics performance and is positively correlated with students' achievement because HSES can provide students with a variety of learning resources such as books and tutoring [38]. To a certain extent, the low economic conditions limit the academic improvement of LSES college students. The results imply that the mental health of LSES college students has a significant predictive effect on academic achievement. When considering the external factors of academic achievement, it is necessary to focus on internal psychological mechanism among LSES college students.

### 4.3. Mediating Role of Social Support between Mental Health and Academic Achievement

We discover that social support (significant other support, family support, and friend support) is significantly positively correlated with GPA. More recent studies have found that the more social support provided by teachers, the higher academic achievement of students is [39]. Parental support helps students form good study habits and well-being, thereby improving students' academic achievement [40]. Similarly, peer support also had a significant predictive effect on students' academic achievement. Such as students who receive more peer support will be more confident and devote more time and energy to learning [41]. Active social support is conducive to improving students' learning efficiency and self-confidence to improving learning motivation and academic achievement [42].

The current study showed the mediating role of social support in the relationship between mental health and GPA, which indicates that the HSES, the higher students' perceived social support level, and perceived social support can further improve students' level of learning outcomes [43]. Parental involvement plays an intermediary role between SES and academic achievement. On the contrary, improper parental support can lead to a decrease in academic achievement. For instance, if parents are over-involved in supervision and control, it will lead to a decrease in students' academic achievement [44]. A study in 2018 among 413 adolescents in the United States found that family social support mediated students' depression and academic achievement; the higher the social support, the lower the depression level and the better academic achievement [45]. A recent study in the United States in 2020 found that peer social support and social engagement performed a mediating role between adolescents' social anxiety and academic achievement; socially anxious adolescents receive less peer support, which will lead to lower social engagement and poor academic achievement [46]. As discussed, if students with poor mental health cannot actively seek social support, their academic achievement will be further affected.

## 5. Limitations

A few limitations need to be considered for the study. First, it should be noted that this study has examined several self-rating scales through online questionnaires because of epidemic situation, and we performed our survey between May and June 2020, so the results may be biased due to the subject's response bias. Moreover, the study did not do the differences between males and females; thus, it is necessary to conduct research on subjects of different genders in the future studies and conduct investigations in normal period. Finally, because the study only selected some students from one university of Shaanxi province in China, the sample representativeness needs to be considered in the future. Relevant research can add sampling from other regions, and gender differences and other relevant influencing factors need to be further analyzed.

## 6. Conclusion

In conclusion, the present study sheds light on the relationship between mental health and GPA among the LSES college students compared to HSES. The results verify that mental health can significantly affect the individual's academic achievement, and social support has a mediate role between mental health and GPA. It shows that LSES students, especially those with a poor mental health, need social support. This research has a lot of practical implications. First, it may help campus administrators and health providers more effectively identify the LSES students at high risk for mental illness. Second, educators are supposed to guide students' study from external behavior and pay more attention to the shaping of inner mental health level. Moreover, the government, society, school, and family should help LSES students to establish a positive social network and actively seek social support, to improve their academic achievement and mental health.

## Figures and Tables

**Figure 1:** The hypothesized model of mental health, GPA, and social support.

**Figure 2:** The mediation model with social support as mediators. ^*∗*^*p* < 0.05, ^*∗∗*^*p* < 0.01, and ^*∗∗∗*^*p* < 0.001.

**Table 1:** Clinical variables in LSES and HSES groups (*N* = 1141).

Variables	LSES (*N* = 640)	HSES (*N* = 501)	T	*p*
	Mean (sd)	Mean (sd)		
State anxiety	40.164 (9.163)	38.607 (9.692)	2.777	0.006
Trait anxiety	40.842 (8.600)	39.471 (9.007)	2.618	0.009
Self-esteem	17.014 (3.659)	18.395 (4.359)	−5.816	0.000
Depression	7.153 (6.520)	5.886 (6.098)	3.351	0.001
Internet addiction	41.288 (11.439)	37.749 (11.576)	5.159	0.000
Significant other support	19.222 (5.316)	20.653 (5.241)	−4.540	0.000
Family support	20.219 (5.147)	21.253 (5.277)	−3.333	0.001
Friend support	21.291 (4.467)	22.359 (4.120)	−4.149	0.000
GPA	2.686 (0.671)	2.991 (0.682)	−7.567	0.000

Note: ^*∗*^*p* < 0.05, ^*∗∗*^*p* < 0.01, and ^*∗∗∗*^*p* < 0.001.

**Table 2:** Descriptive statistics and correlations of all variables.

	Mean	SD	1	2	3	4	5	6	7	8	9
1. State anxiety	39.480	9.427	1								
2. Trait anxiety	40.240	8.804	0.762^*∗∗*^	1							
3. Self-esteem	17.621	4.038	−0.394^*∗∗*^	-0.424^*∗∗*^	1						
4. Depression	6.597	6.366	0.607^*∗∗*^	0.622^*∗∗*^	−0.508^*∗∗*^	1					
5. Internet addiction	39.734	11.628	0.304^*∗∗*^	0.330^*∗∗*^	−0.510^*∗∗*^	0.403^*∗∗*^	1				
6. Significant other support	19.850	5.328	−0.576^*∗∗*^	−0.602^*∗∗*^	0.419^*∗∗*^	−0.517^*∗∗*^	−0.388^*∗∗*^	1			
7. Family support	20.673	5.228	−0.559^*∗∗*^	−0.576^*∗∗*^	0.419^*∗∗*^	−0.579^*∗∗*^	−0.354^*∗∗*^	0.741^*∗∗*^	1		
8. Friend support	21.760	4.348	−0.428^*∗∗*^	−0.441^*∗∗*^	0.389^*∗∗*^	−0.503^*∗∗*^	−0.310^*∗∗*^	0.626^*∗∗*^	0.705^*∗∗*^	1	
9. GPA	2.820	0.692	−0.619^*∗∗*^	−0.597^*∗∗*^	0.466^*∗∗*^	−0.570^*∗∗*^	−0.413^*∗∗*^	0.617^*∗∗*^	0.609^*∗∗*^	0.550^*∗∗*^	1

Note: ^*∗*^*p* < 0.05, ^*∗∗*^*p* < 0.01, and ^*∗∗∗*^*p* < 0.001.

**Table 3:** Bootstrapping indirect effects and 95% confidence interval for the model pathways.

Paths	BootEffect	Bootse	Boot lower bounds	Boot upper bounds
State anxiety⟶significant other support⟶GPA	−0.009	0.001	−0.011	−0.006
State anxiety⟶family support⟶GPA	−0.006	0.001	−0.008	−0.003
State anxiety⟶friend support⟶-GPA	−0.006	0.001	−0.007	−0.004
Trait anxiety⟶significant other support⟶GPA	−0.010	0.001	−0.013	−0.008
Trait anxiety⟶family support⟶GPA	−0.007	0.001	−0.010	−0.004
Trait anxiety⟶friend support⟶GPA	−0.006	0.001	−0.008	−0.004
Self-Esteem⟶significant other support⟶GPA	0.021	0.002	0.016	0.025
Self-Esteem⟶family support⟶GPA	0.015	0.003	0.010	0.020
Self-Esteem⟶friend support⟶GPA	0.010	0.002	0.006	0.014
Depression⟶significant other support⟶GPA	−0.016	0.002	−0.020	−0.013
Depression⟶family support⟶GPA	−0.009	0.002	−0.014	−0.005
Depression⟶friend support⟶GPA	−0.007	0.002	−0.011	−0.004
Internet addiction⟶significant other support⟶GPA	−0.007	0.001	−0.008	−0.005
Internet addiction⟶family support⟶GPA	−0.005	0.001	−0.006	−0.003
Internet addiction⟶friend support⟶GPA	−0.003	0.001	−0.004	−0.002

*Note.* BootEffect, standardized indirect effect; Bootse, bootstrap standard errors; ^*∗*^*p* < 0.05, ^*∗∗*^*p* < 0.01, and ^*∗∗∗*^*p* < 0.001.

## Data Availability

All data, models, and code generated or used during the study are provided within the article article.
